# Correlation between Ultrasonographic Appearance of Papillary Thyroid Microcarcinoma and BRAF V600E Mutation

**DOI:** 10.1155/2022/5916379

**Published:** 2022-03-21

**Authors:** Songnian Liang, Kun Huang

**Affiliations:** ^1^Department of Radiology, The First Affiliated Hospital of China Medical University, Shenyang, Liaoning, China; ^2^Department of Ultrasonic Diagnosis, The First Affiliated Hospital of China Medical University, Shenyang, Liaoning, China

## Abstract

The study was conducted to investigate the correlation between the ultrasonographic appearance of a thyroid nodule and the BRAF V600E mutation. Patients with thyroid nodules (*n* = 186), for which BRAF V600E testing and cytopathology analysis were performed, and who underwent subsequent surgery for nodule resection were enrolled in this study. For each patient, color Doppler ultrasonography was performed to observe the variables of the nodules. The nodules were then characterized using the thyroid imaging reporting and data system classification TI-RADS. Furthermore, the ultrasonographic appearance of the control group, encompassing patients with nodular thyroid goiters, and the case group, encompassing patients with papillary thyroid microcarcinoma (PTMC), was statically analyzed. Similarly, a statistical analysis of the ultrasonographic appearance of the BRAF V600E-positive and BRAF V600E-negative subgroups was also performed. The accuracy was significantly different for the corresponding values when color Doppler ultrasonography, BRAF V600E testing, or cytopathology alone was used for diagnosis. There were significant differences in the ultrasonographic appearance variables between the control and case groups. Comparing with the BRAF V600E-negative subgroup of the case group, the ultrasonographic appearances of the BRAF V600E-positive subgroup showed less circumscribed and more irregularly shaped nodules, with significantly different aspect ratios of >1. The combination of BRAF V600E testing and color Doppler ultrasonography or cytopathology improved the accuracy of the PTMC diagnose. We found that the ultrasonographic appearance of thyroid nodules was related to PTMC.

## 1. Introduction

Thyroid carcinoma is the most common malignant tumor of the endocrine system, and it has been increasingly studied by clinicians and researchers. In the past years, its incidence has gradually increased, with the fastest increase observed among all types of malignant tumors [1]. Specifically, in terms of pathological type of thyroid carcinoma, there has been a growing incidence of papillary carcinoma, while in terms of pathological stage microcarcinoma has exhibited the fastest increase in incidence [2, 3]. According to the latest SEER statistics, nearly 90% of thyroid carcinomas are papillary carcinomas [4], reinforcing the importance of studying papillary thyroid microcarcinoma (PTMC). In addition, microcarcinoma has a high cervical lymph node metastasis rate of 30–70% [5–7]. Some patients with microcarcinoma have local recurrences very soon after surgery or can even present initially with distant metastases to the lungs or bones [8, 9]. Therefore, the present study is aimed at assessing the risk of PTMC by exploring the ultrasonographic appearance of thyroid nodules.

Many thyroid carcinomas, mainly follicular cell-derived thyroid carcinomas, are caused by genetic mutations, through effects on molecular signaling pathways like MAPK and PI3K/AKT. The most commonly found mutated genes include *BRAF*, *H-RAS*, *K-RAS*, *N-RAS*, and *PTEN*. The BRAF V600E mutation is the most common in papillary thyroid carcinoma (PTC) [10], corresponding to 28–83% of all gene mutations observed and accounting for about 90% of all *BRAF* mutations [11–13]. However, it has not been found in normal thyroid tissues or benign lesions [14–18]. In addition, the BRAF V600E mutation is closely related to recurrence of papillary carcinomas and patient death. Therefore, the main objective of this study was to investigate PTMC and evaluate the correlation between its ultrasonographic appearance and the *BRAF* gene. According to the World Health Organization (WHO), a PTC with a maximum tumor diameter < 1.0 cm is considered a PTMC [13, 19, 20]. As defined by WHO in the 2004 edition of the Tumor Pathology and Genetics of Endocrine Organs, microcarcinoma is a subtype of thyroid carcinoma, and thyroid microcarcinoma is only referred to as a PTMC [21]. Therefore, all thyroid microcarcinomas examined in this study were PTMC.

## 2. Material and Methods

### 2.1. Research Subjects

This study was approved by the Ethics Committee of China Medical University. Informed consent was obtained from all patients enrolled after full explanation of the purpose and nature of all procedures performed.

The study included 186 patients presenting thyroid nodules with a maximum diameter of <1.0 cm, for which preoperative BRAF V600E testing and cytopathology analysis were performed, and who underwent subsequent surgery to remove thyroid nodules at the Department of Thyroid Surgery of the First Affiliated Hospital of China Medical University from January 2017 to March 2018. None of the patients had surgical contraindications. The patients were aged 19–70 years, mean age of 38.6 ± 2.7 years, and included 143 females and 43 males. There were 100 pathologically diagnosed cases of PTMC, 80 cases of nodular goiters, and 6 cases of follicular thyroid carcinomas. All PTMC were solitary nodules. The diameters of PTMCs and nodular goiters were in the range of 0.5–1.0 cm, while nodules with diameters of less than 0.5 cm were excluded from this study. Additionally, the patients with two nodules were also excluded.

### 2.2. Procedures

Color Doppler ultrasound diagnostic apparatuses (Aixplorer, Supersonic Imagine, France; EPIQ7, Philips, USA) with probe frequencies of 5–12 MHz were used. The subjects were scanned in the supine position for thyroid gland to determine the size, number, location, internal echo, border, morphology, and blood flow of thyroid nodules; the nodules were examined to determine if their aspect ratios were >1 and if they had had cystic change, microcalcification, and/or attenuation. Moreover, the elasticity modulus values were measured and the nodules were classified according to TI-RADS. Before surgery, each module was subjected to fine needle aspiration for BRAF V600E testing and cytopathology analysis. The pathological diagnosis was conducted after nodular surgery. The nodule locations were classified as either in the central or peripheral regions, where the peripheral region included the isthmus and anterior, posterior, lateral, and medial margins.

Regarding the method to measure the elasticity modulus values, we used the Shear Wave Elastography (SWE) mode, in which the elastic range was set to 180 kPa, the diameter of the elasticity value measurement area was set to 5.0 mm, and the sampling frame was uniformly filled with color. During each measurement, patients were requested to hold their breath for 3–5 s, and, when stabilized, the images were stored as frames. Meanwhile, two-dimensional and elasticity images (with color coding in the range of 0–180 kPa) were displayed to determine the range and position of the region of interest (ROI) within the selected mass. Subsequently, the ROI elasticity modulus values were calculated, including the mean and minimum and maximum values in kPa. Each nodule was measured in triplicate and the results were averaged. Each patient was examined by the same methods, and the BRAF V600E testing was performed by the Amplification Refractory Mutation System (ARMS) method.

Patients with PTMC and nodular goiters were designated as the case and control groups, respectively. To diagnose thyroid nodules by either color Doppler ultrasonography, BRAF V600E testing, or cytopathology alone or by the latter two methods combined, we calculated the specificity, sensitivity, accuracy, and positive and negative predictive values; the accuracy was then statistically analyzed. Ultrasonographic appearance variables of the nodules (location, border, internal echo, morphology, microcalcification, aspect ratio > 1, attenuation, cystic change, blood flow, and elasticity modulus value) and patient age and gender were statistically compared between the two groups. The case group was further divided into two subgroups according to the BRAF V600E testing results (positive or negative). The ultrasonographic appearance variables of the nodules and patient age and gender in each subgroup were analyzed statistically to determine whether there was a correlation with BRAF V600E.

The thyroid nodules were diagnosed as benign and malignant using color Doppler ultrasonography based on the following criteria: the nodules of TI-RADS grades 3 and 4a were benign, while those of TI-RADS grades 4b, 4c, and 5 were malignant. The thyroid nodules were diagnosed as malignant or benign using BRAF V600E testing based on the following criteria: the nodules positive for BRAF V600E were malignant, while those that were negative were benign.

Each patient was examined using the same method, supervised by at least two physicians, both being associate professors, who reached an agreement through discussion in the case of controversy.

### 2.3. Statistical Analysis

Statistical analysis was performed with SPSS software version 19.0, and measurement data were expressed as the mean ± standard deviation. The specificity, sensitivity, accuracy, and positive and negative predictive values were calculated. Chi-square tests were used to compare the ultrasonographic appearance of thyroid nodules between the case and control groups and between the BRAF V600E-positive and BRAF V600E-negative subgroups of the case group. Univariate and multivariate analyses were performed by Cox proportional hazards regression models to estimate HR and 95% CI.

## 3. Results

The control group consisted of 80 patients, of whom 16 were diagnosed with thyroid nodules of TI-RADS grade 3, 46 of grade 4a, and 18 of grade 4b, according to the color Doppler ultrasonography. The BRAF V600 testing results of these thyroid nodules were all negative (Figures 1(a)–1(f)); and the cytopathology analysis diagnosed 6 cases of malignant nodules and 64 of benign, with 10 diagnostically uncertain cases. The case group consisted of 100 patients, of whom 15 were diagnosed with thyroid nodules of TI-RADS grade 4a, 67 of grade 4b, and 18 of grade 4c, according to the color Doppler ultrasonography. The BRAF V600 testing of the thyroid nodules showed positive results for 56 patients, while it was negative for 44 patients (Figures 1(a)–1(f)). The cytopathology analysis diagnosed 61 cases of malignant nodules and 28 of benign, with 11 diagnostically uncertain cases.

The color Doppler ultrasonography of the thyroid nodules alone exhibited specificity of 77.5%, sensitivity of 85%, accuracy of 81.67%, positive predictive value of 82.52%, and negative predictive value of 80.52%. Diagnosis of the nodules by BRAF V600E testing alone showed specificity of 100%, sensitivity of 56%, accuracy of 75.56%, positive predictive value of 100%, and negative predictive value of 64.52%. Diagnosis of the nodules by cytopathology analysis alone showed specificity of 91.43%, sensitivity of 68.54%, accuracy of 78.62%, positive predictive value of 90.04%, and negative predictive value of 69.57%. The combination of color Doppler ultrasonography and *BRAF* V600E testing showed specificity of 77.5%, sensitivity of 96%, accuracy of 87.78%, positive predictive value of 84.21%, and negative predictive value of 93.94%. The combination of *BRAF* V600E testing and cytopathology analysis showed specificity of 91.43%, sensitivity of 86.46%, accuracy of 88.55%, positive predictive value of 93.26%, and negative predictive value of 83.12%.

There was no significant difference (*P* > 0.05) in the accuracy of the PMTC diagnosis among color Doppler ultrasonography, BRAF V600E testing, and cytopathology analysis. However, each of the three methods, when used alone, was significantly different (*P* < 0.05) from their combinations in terms of accuracy of PMTC diagnosis, as shown in Table 1.

There was a statistically significant difference (*P* < 0.05) between the case and control groups for some of the Doppler ultrasonographic appearance variables, including unclear border, hypoechogenicity, irregular morphology, microcalcification, attenuation, cystic change, and elasticity modulus value. However, there was no statistical difference in location, gender, age, aspect ratio > 1, or blood flow type (*P* > 0.05) between the two groups, as shown in Table 2.

The univariate analysis showed that the PTMC was correlated with border echo, internal echo, morphology, microcalcification, aspect ratio, attenuation, cystic change, and elasticity modulus value. Further, the multivariate Cox regression analysis showed that the border echo (HR = 6.812, 95%CI = 2.897–16.016, *P* < 0.001), internal echo (HR = 7.977, 95%CI = 3.211–19.817, *P* < 0.001), morphology (HR = 6.154, 95%CI = 2.687–14.095, *P* < 0.001), microcalcification (HR = 6.768, 95%CI = 2.835–16.159, *P* < 0.001), attenuation (HR = 0.208, 95%CI = 0.076–0.572, *P* = 0.002), cystic change (HR = 7.313, 95%CI = 2.521–21.211, *P* < 0.001), and elasticity modulus value (HR = 3.074, 95%CI = 1.369–6.901, *P* = 0.006) were independent predictors for diagnosis of PTMC (Table 3).

There was a statistically significant difference (*P* < 0.05) between the BRAF V600E-positive and BRAF V600E-negative subgroups for some of the color Doppler ultrasonographic variables, namely, unclear border, irregular morphology, and aspect ratio > 1. However, there was no statistical difference (*P* > 0.05) for the other variables (location, gender, age, echo, microcalcification, attenuation, cystic change, blood flow type, and elasticity modulus value) between the two subgroups, as shown in Table 4.

The univariate analysis showed that the BRAF V600E mutation was correlated with border echo, morphology, aspect ratio, attenuation, and elasticity modulus value. Further, the multivariate Cox regression analysis showed that the border echo (HR = 17.889, 95%CI = 3.674–87.093, *P* < 0.001), morphology (HR = 0.07, 95%CI = 0.012–0.414, *P* = 0.003), and aspect ratio (HR = 23.476, 95%CI = 4.555–121.004, *P* < 0.001) were independent predictors for BRAF V600E mutation (Table 5).

## 4. Discussion

The progression of PTMC is rapid, and its incidence has significantly increased in recent years. Despite controversy over PTMC surgery, its metastasis to the central lymph nodes is indisputable, occurring at a high rate of 24–64%. Moreover, PTMC has high recurrence and mortality rates [22, 23]. Therefore, a high diagnostic accuracy is necessary in clinical settings, as surgery is the commonly accepted method of treating metastatic PMTC. However, currently, the diagnostic accuracy of PTMC is not high, and missed diagnoses and misdiagnoses occur frequently. At present, the main diagnostic method is color Doppler ultrasonography with an accuracy of 75–90% [24].

Recently, with the advances in molecular biology technology, rapid developments have occurred in the field of biomolecular research on thyroid carcinoma. As a research hotspot in recent years, the BRAF V600E mutation has become a new prospect for the early detection of PTMC. In fact, the *BRAF* V600E allele is an oncogene for thyroid carcinoma. However, the sensitivity of BRAF V600E testing is very low (reaching only 45%), while its specificity is as high as 99.5% [13, 25–27]. Moreover, Li et al. [13, 28] reported that the BRAF V600E mutation is closely related to extracapsular invasion of PTC, lymph node metastasis, and high TNM stage, leading to a higher capsular invasion rate ^29^. PTCs with the BRAF V600E mutation are highly invasive and prone to infiltrate the tissues surrounding the thyroid gland, leading to late clinical staging [28–30] and worse prognosis [29, 31, 32]. Therefore, obtaining positive BRAF V600E testing results is a pivotal step for diagnosis. In this study, the BRAF V600E testing results and the ultrasonographic appearance of the thyroid nodules were combined to increase the accuracy of PTMC diagnosis, allowing the invasiveness of nodules to be inferred. With this combination, PTMC can be detected in a more reasonable manner to identify the nodules that are susceptible to metastasis.

In agreement with the literature [23, 25, 27], our findings revealed 100% specificity and 56% sensitivity for the *BRAF* V600E testing. This specificity rate means that patients positive for BRAF V600E are diagnosed with PTC without misdiagnoses. Therefore, positive results in BRAF V600E testing are of great value. However, the very low diagnostic sensitivity results in many missed diagnoses of PTC. Considering this, it is necessary to seek new markers to evaluate thyroid carcinoma. The statistical difference found between the combination of BRAF V600E testing with color Doppler ultrasonography or cytopathology and either method alone indicated that the combined diagnosis compensated for the limitations of the methods individually (i.e., the low sensitivities of BRAF V600E testing and cytopathology and the low specificity of color Doppler ultrasonography), thereby greatly enhancing the accuracy of PTMC detection and greatly reducing the proportion that cannot be determined by cytopathology analysis. For nodules that cannot be defined or tend to be benign by cytopathology analysis, once a positive result for BRAF V600E testing is determined, the nodule would be diagnosed as malignant. Therefore, BRAF V600E testing is a good auxiliary means for improving the diagnosis rate of thyroid nodules ^34^.

Statistically significant differences were observed in some of the ultrasonographic appearance variables (unclear border, hypoechogenicity, irregular morphology, microcalcification, attenuation, cystic change, and elasticity modulus value) between the control and case groups, indicating that these variables can be considered specific manifestations of thyroid malignant nodules, consistent with previously reported findings [33]. PTMC nests are not susceptible to liquefied necrosis, and cystic change is rarely seen, while they have a tendency to undergo longitudinal division. Therefore, irregular morphologies, unclear borders, and nodular attenuation are more likely to occur in microcarcinomas. However, there is no statistical difference in aspect ratios > 1, which is inconsistent with the research results of other scholars. The main reason is that the object of this study is nodules with a maximum diameter of less than 1 cm, and the number of cases is relatively small. Among them, the proportion of malignant nodules with an aspect ratio greater than 1 is not significantly higher than that of benign nodules.

In this study, the presence of unclear borders, irregular morphologies, and aspect ratios > 1 in the ultrasonographic appearance of the BRAF V600E-positive subgroup was significantly more common than in that of the negative group. This is also consistent with the findings of Skubisz et al. [34]. Malignant nodules with irregular morphologies are prone to mutations, meaning that it is necessary to pay attention to irregular morphologies when evaluating and classifying nodules. Moreover, unclear borders are usually accompanied by aspect ratios > 1. If such a nodule is suspected to be malignant, it should be surgically removed to prevent lymph node metastasis, because the probability that its oncogene test result will be positive is greatly increased, compared to more regular nodules. An explanation for the statistically significant difference in ultrasonographic appearance is that the cells of cancer nodules grow and are arranged in a longitudinal manner; in the early stages of thyroid carcinoma, the cancer cells in the anterior and posterior sides of the tumor undergo division, while those growing in other directions are at a relatively quiescent phase. This difference results in longer radial extension of the tumor in the anterior and posterior directions than in the right and left directions—a growth pattern totally contrasting with that of benign nodules [35]. In addition, the malignancy assessed by ultrasound was not obvious for six patients, but the *BRAF* V600E testing was positive, and surgery was not performed immediately. After one year, the nodule increased significantly and the anteroposterior diameter exceeded 1.0 cm, accompanied by lymph node metastasis. Therefore, BRAF V600E expression was positive and tumor invasiveness could be related [36, 37]. Further research is needed for future follow-up.

The diameter of the nodules selected in this study was between 0.5 and 1.0 cm, mainly because the study was primarily focused on papillary microcarcinomas (which have diameters < 1.0 cm). Additionally, the minimum diameter of the nodules investigated in the case group was 0.5 cm, primarily because examining smaller nodules would allow even smaller cancer nests to be used for BRAF V600E testing via fine needle aspiration, resulting in a higher false-negative rate.

Regarding the limitations of this study, as BRAF V600E testing in our hospital is performed relatively late and no large sample size was collected, a larger sample is needed to verify further our conclusions. Moreover, one patient with multiple nodules was excluded from the study and thus was not subjected to ultrasonographic analysis.

In conclusion, the combined application of BRAF V600E testing and color Doppler ultrasonography or cytopathology can improve the accuracy of PTMC diagnosis. Among the ultrasonographic observations of thyroid nodules, unclear borders, hypoechogenicity, irregular morphologies, microcalcification, attenuation, the absence of cystic change, and the elasticity modulus value can be used in combination as indicators to distinguish between benign and malignant nodules. For malignant nodules, ultrasonographic appearances with unclear borders, irregular morphologies, and aspect ratios > 1 were associated with positive results of BRAF V600E testing, suggesting that such nodules are prone to metastasis and are associated with poor prognosis. This correlative study of ultrasonographic appearances of thyroid nodules may represent a scientific foundation for artificial intelligence-based ultrasonographic diagnosis of thyroid carcinoma.

## Figures and Tables

**Figure 1:** Ultrasonography of thyroid nodules. (a, b) Ultrasonographic appearance of a thyroid nodule pathologically diagnosed as a nodular thyroid goiter showing hypoechogenicity, unclear borders. (c, d) Ultrasonographic appearance of a thyroid nodule pathologically diagnosed as PTMC and negative for the BRAF V600E mutation, showing hypoechogenicity and central blood flow. (e, f) Ultrasonographic appearance of a thyroid nodule pathologically diagnosed with PTMC and positive for the BRAF V600E mutation, showing hypoechogenicity, unclear borders, and aspect ratios > 1.

**Table 1:** PTMC diagnostic results obtained via color Doppler ultrasonography, BRAF V600E testing, or cytopathology analysis alone and in combination, versus the pathological results.

	Classification	Pathology (number of cases)		Accuracy	*P* value^∗^
		M	B		
(1) Color Doppler ultrasonography	M	85	18	81.67%	>0.05
	B	15	62		

(2) BRAF V600E testing	M	56	0	75.56%	>0.05
	B	44	80		

(3) Cytopathology analysis	M	61	6	78.62%	>0.05
	B	28	64		

	Uncertain	11	10		

Combination of (1) and (2)	M	96	18	87.78%	<0.05
	B	4	62		

Combination of (2) and (3)	M	83	6	88.55%	<0.05
	B	13	64		

	Uncertain	4	10		

^∗^ *P* < 0.05: statistically different; *P* > 0.05: not statistically different; M: malignant nodule; B: benign nodule.

**Table 2:** Correlation between the ultrasonographic appearances of PTMC and nodular thyroid goiter.

Factor	Number of cases	Pathological expression		*P* value^∗^
		PTMC positive	PTMC negative	
Location				
Marginal region or near isthmus	131	69	62	0.194
Central region	49	31	18	
Gender				
Female	140	82	58	0.128
Male	40	18	22	
Age (years)				
≥45	97	51	46	0.385
<45	83	49	34	
Border echo				
Unclear	96	68	28	<0.001^∗^
Clear	84	32	52	
Internal echo				
Hypoechoic	152	92	60	0.002^∗^
Hyperechoic	28	8	20	
Morphology				
Irregular	112	80	32	<0.001^∗^
Regular	68	20	48	
Microcalcification				
Yes	136	84	52	0.003^∗^
No	44	16	28	
Aspect ratio				
>1	56	36	20	0.113
<1	124	64	60	
Attenuation				
Yes	36	12	24	0.003^∗^
No	144	88	56	
Cystic change				
No	152	96	56	<0.001^∗^
Yes	28	4	24	
Blood flow				
Central	64	36	28	
Marginal	116	64	52	0.889
Elasticity modulus value				
>63 kPa	89	60	29	0.002^∗^
<63 kPa	91	40	51	

^∗^ *P* < 0.05: statistically different; *P* > 0.05: not statistically different.

**Table 3:** Univariate and multivariate Cox regression of ultrasonographic appearances for PTMC.

	Univariate analysis		Multivariate analysis	
	HR (95% CI)	*P* value	HR (95% CI)	*P* value
Location	0.617 (0.315~1.208)	0.159	—	—
Gender	1.728 (0.851~3.507)	0.130	—	—
Age (years)	0.903 (0.499~1.635)	0.737	—	—
Border echo	4.333 (2.313~8.118)	<0.001^∗^	6.812 (2.897~16.016)	<0.001^∗^
Internal echo	2.697 (1.205~6.034)	0.016^∗^	7.977 (3.211~19.817)	<0.001^∗^
Morphology	4.500 (2.381~8.503)	<0.001^∗^	6.154 (2.687~14.095)	<0.001^∗^
Microcalcification	2.629 (1.312~5.269)	0.006^∗^	6.768 (2.835~16.159)	<0.001^∗^
Aspect ratio	3.392 (1.417~8.121)	0.006^∗^	2.054 (0.862~4.894)	0.104
Attenuation	0.412 (0.199~0.853)	0.017^∗^	0.208 (0.076~0.572)	0.002^∗^
Cystic change	4.929 (2.072~11.721)	<0.001^∗^	7.313 (2.521~21.211)	<0.001^∗^
Blood flow	1.091 (0.591~2.014)	0.781	—	—
Elasticity modulus value	2.638 (1.438~4.838)	0.002^∗^	3.074 (1.369~6.901)	0.006^∗^

^∗^ *P* < 0.05: statistically different; *P* > 0.05: not statistically different.

**Table 4:** Correlation between the ultrasonographic appearance of PTMC and the BRAF V600E mutation.

Factor	Number of cases	BRAF V600E mutation		*P* value^∗^
		Positive	Negative	
Location				
Marginal region or near isthmus	68	38	30	0.972
Central region	32	18	14	
Gender				
Female	82	47	35	0.571
Male	18	9	9	
Age (years)				
≥45	55	34	21	0.195
<45	45	22	23	
Border echo				
Unclear	70	49	21	<0.001^∗^
Clear	30	7	23	
Internal echo				
Hypoechoic	89	48	41	0.236
Hyperechoic	11	8	3	
Morphology				
Irregular	75	35	40	0.001^∗^
Regular	25	21	4	
Microcalcification				
Yes	83	45	38	0.427
No	17	11	6	
Aspect ratio				
>1	36	30	6	0.001^∗^
<1	64	26	38	
Attenuation				
Yes	14	11	3	0.067
No	86	45	41	
Cystic change				
No	92	49	43	
Yes	8	7	1	0.061
Blood flow				
Central	37	18	19	0.256
Marginal	63	38	25	
Elasticity modulus value				
>63 kPa	58	37	21	0.065
<63 kPa	42	19	23	

^∗^ *P* < 0.05: statistically different; *P* > 0.05: not statistically different.

**Table 5:** Univariate and multivariate Cox regression of ultrasonographic appearances for BRAF V600E mutation.

	Univariate analysis		Multivariate analysis	
	HR (95% CI)	*P* value	HR (95% CI)	*P* value
Location	0.985 (0.422~2.297)	0.972	—	—
Gender	1.343 (0.483~3.733)	0.572	—	—
Age (years)	1.693 (0.762~3.761)	0.196	—	—
Border echo	7.667 (2.853~20.602)	<0.001^∗^	17.889 (3.674~87.093)	<0.001^∗^
Internal echo	0.439 (0.109~1.764)	0.246	—	—
Morphology	0.167 (0.052~0.532)	0.002^∗^	0.070 (0.012~0.414)	0.003^∗^
Microcalcification	0.646 (0.218~1.910)	0.430	—	—
Aspect ratio	7.308 (2.666~20.035)	<0.001^∗^	23.476 (4.555~121.004)	<0.001^∗^
Attenuation	6.668 (1.299~34.241)	0.023^∗^	2.079 (0.345~12.541)	0.425
Cystic change	0.163 (0.019~1.377)	0.096	—	—
Blood flow	0.623 (0.275~1.413)	0.258	—	—
Elasticity modulus value	2.513 (1.105~5.712)	0.028^∗^	1.995 (0.228~17.475)	0.533

^∗^ *P* < 0.05: statistically different; *P* > 0.05: not statistically different.

## Data Availability

Data are available on request from the authors.

## References

[1] Li M., Zhu X. Y., Lv J. (2017). Risk factors for predicting central lymph node metastasis in papillary thyroid microcarcinoma (CN0): a study of 273 resections. *European Review for Medical and Pharmacological Sciences*.

[2] Chen A. Y., Jemal A., Ward E. M. (2009). Increasing incidence of differentiated thyroid cancer in the United States, 1988-2005. *Cancer*.

[3] Sugitani I., Ito Y., Takeuchi D. (2021). Indications and strategy for active surveillance of adult low-risk papillary thyroid microcarcinoma: consensus statements from the Japan Association of Endocrine Surgery task force on management for papillary thyroid microcarcinoma. *Thyroid*.

[4] Davies L., Welch H. G. (2006). Increasing incidence of thyroid cancer in the United States, 1973-2002. *JAMA*.

[5] Lim Y. C., Choi E. C., Yoon Y. H., Kim E. H., Koo B. S. (2009). Central lymph node metastases in unilateral papillary thyroid microcarcinoma. *The British Journal of Surgery*.

[6] Mercante G., Frasoldati A., Pedroni C. (2009). Prognostic factors affecting neck lymph node recurrence and distant metastasis in papillary microcarcinoma of the thyroid: results of a study in 445 patients. *Thyroid*.

[7] Lombardi C. P., Bellantone R., de Crea C. (2010). Papillary thyroid microcarcinoma: extrathyroidal extension, lymph node metastases, and risk factors for recurrence in a high prevalence of goiter area. *World Journal of Surgery*.

[8] Xu Y. H., Song H. J., Qiu Z. L., Luo Q. Y. (2011). Brain metastases with exceptional features from papillary thyroid carcinoma: report of three cases. *Hellenic Journal of Nuclear Medicine*.

[9] Varsavsky M., Cortés B. M., Alonso G., García M. A., Muñoz T. M. (2011). Metastatic adenopathy from a thyroid microcarcinoma: final diagnosis of a presumed paraganglioma. *Endocrinología y nutrición: órgano de la Sociedad Española de Endocrinología y Nutrición*.

[10] Xing M., Westra W. H., Tufano R. P. (2005). BRAF mutation predicts a poorer clinical prognosis for papillary thyroid cancer. *The Journal of Clinical Endocrinology and Metabolism*.

[11] Kim S. W., Lee J. I., Kim J. W. (2010). BRAFV600E mutation analysis in fine-needle aspiration cytology specimens for evaluation of thyroid nodule: a large series in aBRAFV600E-Prevalent population. *The Journal of Clinical Endocrinology and Metabolism*.

[12] Min H. S., Lee C., Jung K. C. (2013). Correlation of immunohistochemical markers and BRAF mutation status with histological variants of papillary thyroid carcinoma in the Korean population. *Journal of Korean Medical Science*.

[13] Kwak J. Y., Kim E. K., Chung W. Y., Moon H. J., Kim M. J., Choi J. R. (2009). Association of BRAFV600EMutation with poor clinical prognostic factors and US features in Korean patients with papillary thyroid microcarcinoma. *Radiology*.

[14] Millington G. W. (2013). Mutations of theBRAFgene in human cancer, by Davieset al. (Nature2002; 417: 949-54). *Clinical and Experimental Dermatology*.

[15] DeLuca A. M., Srinivas A., Alani R. M. (2008). BRAF kinase in melanoma development and progression. *Expert reviews in Molecular Medicine*.

[16] Liu Z., Lv T., Xie C., Di Z. (2018). *BRAF* V600E Gene Mutation Is Associated With Bilateral Malignancy of Papillary Thyroid Cancer. *The American Journal of the Medical Sciences*.

[17] Kebebew E., Weng J., Bauer J. (2007). The prevalence and prognostic value of BRAF mutation in thyroid cancer. *Annals of Surgery*.

[18] Kim T. H., Park Y. J., Lim J. A. (2012). The association of the BRAFV600E mutation with prognostic factors and poor clinical outcome in papillary thyroid cancer. *Cancer*.

[19] Sobin L. H. (1990). Histological typing of thyroid tumours. *Histopathology*.

[20] Shen R., Liyanarachchi S., Li W. (2012). MicroRNA signature in thyroid fine needle aspiration cytology applied to "atypia of undetermined significance" cases. *Thyroid*.

[21] DeLellis R. A. (2011). Parathyroid tumors and related disorders. *Modern Pathology*.

[22] Huang X. P., Ye T. T., Zhang L. (2018). Sonographic features of papillary thyroid microcarcinoma predicting high- volume central neck lymph node metastasis. *Surgical Oncology*.

[23] Ferris R. L., Baloch Z., Bernet V. (2015). American Thyroid Association statement on surgical application of molecular profiling for thyroid nodules: current impact on perioperative decision making. *Thyroid*.

[24] Sheth S. (2010). Role of ultrasonography in thyroid disease. *Otolaryngologic clinics of North America*.

[25] Xing M. (2013). Molecular pathogenesis and mechanisms of thyroid cancer. *Nature reviews. Cancer*.

[26] Li F., Chen G., Sheng C. (2015). BRAFV600E mutation in papillary thyroid microcarcinoma: a meta-analysis. *Endocrine-Related Cancer*.

[27] Cooper D. S., Doherty G. M., Haugen B. R. (2009). Revised American Thyroid Association management guidelines for patients with thyroid nodules and differentiated thyroid cancer. *Thyroid*.

[28] Kim M., Bae J. S., Lim D. (2014). Quantification of BRAF V600E alleles predicts papillary thyroid cancer progression. *Endocrine-Related Cancer*.

[29] Xing M., Alzahrani A. S., Carson K. A. (2013). Association between BRAF V600E mutation and mortality in patients with papillary thyroid cancer. *JAMA*.

[30] Lin K. L., Wang O. C., Zhang X. H., Dai X. X., Hu X. Q., Qu J. M. (2010). The BRAF mutation is predictive of aggressive clinicopathological characteristics in papillary thyroid microcarcinoma. *Annals of Surgical Oncology*.

[31] Miccoli P., Basolo F. (2014). BRAF mutation status in papillary thyroid carcinoma: significance for surgical strategy. *Langenbeck's Archives of Surgery*.

[32] Durante C., Puxeddu E., Ferretti E. (2007). BRAF mutations in papillary thyroid carcinomas inhibit genes involved in iodine metabolism. *The Journal of Clinical Endocrinology and Metabolism*.

[33] Li B., Zhang Y., Yin P., Zhou J., Jiang T. (2016). Ultrasonic features of papillary thyroid microcarcinoma coexisting with a thyroid abnormality. *Oncology Letters*.

[34] Skubisz K., Januszkiewicz-Caulier J., Cybula P. (2021). Higher EU-TIRADS-score correlated with BRAF V600E positivity in the early stage of papillary thyroid carcinoma. *Journal of clinical medicine*.

[35] Samir A. E., Vij A., Seale M. K. (2012). Ultrasound-guided percutaneous thyroid nodule core biopsy: clinical utility in patients with prior nondiagnostic fine-needle aspirate. *Thyroid*.

[36] Huang K., Gao N., Bian D., Zhai Q., Yang P., Zhang Y. (2020). Associations of BRAF V600E, clinical pathology and imaging factors with the recurrence rate of papillary thyroid microcarcinoma. *Experimental and Therapeutic Medicine*.

[37] Sezer H., Uren N., Yazici D. (2020). Association between BRAFV600E mutation and the clinicopathological features in incidental papillary thyroid microcarcinoma: a single-center study in Turkish patients. *Northern Clinics of Istanbul*.

